This article has been retracted.

# Inhibition of ZEB1-AS1 confers cisplatin sensitivity in breast cancer by promoting microRNA-129-5p-dependent ZEB1 downregulation

**DOI:** 10.1186/s12935-020-1164-8

**Published:** 2020-03-23

**Authors:** Jin Gao, Yuan Yuan, Lili Zhang, Shaorong Yu, Jianwei Lu, Jifeng Feng, Sainan Hu

**Affiliations:** Department of Medical Oncology, Jiangsu Cancer Hospital, Jiangsu Institute of Cancer Research, The Affiliated Cancer Hospital of Nanjing Medical University, No. 42, Baiziting, Nanjing, 210009 Jiangsu People’s Republic of China

**Keywords:** Long non-coding RNA ZEB1-AS1, ZEB1-AS1/miR-129-5p/ZEB1 signaling pathway, Drug resistance, Breast cancer

## Abstract

**Background:**

Breast cancer is the leading cause of cancer-related mortality in women worldwide. Long non-coding RNAs (lncRNAs) are of critical importance in tumor drug resistance. Herein, this study aims to determine the roles of lncRNA ZEB1-AS1 in drug resistance of breast cancer involving microRNA-129-5p (miR-129-5p) and ZEB1.

**Methods:**

Microarray-based gene expression profiling of breast cancer was conducted to identify the differentially expressed lncRNAs. ZEB1 expression was measured in adjacent and cancerous tissues. Next, MCF-7 and MDA-MB-231 cells were treated with a series of inhibitor, mimic or siRNA to clarify the roles of lncRNA ZEB1-AS1 and miR-129-5p in drug resistance of breast cancer. Then the target relationship of miR-129-5p with lncRNA ZEB1-AS1 and ZEB1 was verified. The expression patterns of miR-129-5p, lncRNA ZEB1-AS1, *Bcl*-*2*, *MDR*-*1*, ZEB1 and corresponding proteins were evaluated. Moreover, the apoptosis and drug resistance of MCF-7 cell were detected by CCK-8 and flow cytometry respectively.

**Results:**

LncRNA ZEB1-AS1 was observed to be an upregulated lncRNA in breast cancer, and ZEB1 overexpression was noted in breast cancerous tissues. MiR-129-5p was revealed to specifically bind to both ZEB1 and lncRNA ZEB1-AS1. Moreover, the expression levels of ZEB1-AS1, ZEB1, *Bcl*-*2*, *MDR*-*1*, and corresponding proteins were decreased, but the expression of miR-129-5p was increased with transfection of miR-129-5p mimic and lncRNA ZEB1-AS1 siRNA. Besides, drug resistance to cisplatin was inhibited, and cell apoptosis was promoted in breast cancer after transfection of miR-129-5p mimic, lncRNA ZEB1-AS1 siRNA, and ZEB1 siRNA.

**Conclusion:**

In conclusion, the study provides evidence that lncRNA ZEB1-AS1 silencing protects against drug resistance in breast cancer by promoting miR-129-5p-dependent ZEB1 downregulation. It may serve as a novel therapeutic target in breast cancer treatment.

## Background

Breast cancer is a common malignancy associated with high mortality rates among women due to a limitation in the clinically proven treatment regimens [1]. Breast cancer is correlated with various extrinsic and intrinsic risk factors, such as environmental and genetic factor, tumor history in direct relatives, late menopause, early menarche and age more than 40 [2]. Reports have exhibited adipocyte secretome to contribute to and facilitate mammary tumor formation, which might provide new insights for the prevention of breast cancer [3]. Anthracyclines and trastuzumab are the extensively used drugs in breast cancer treatment protocol, which induce congestive heart failure as a side effect [4]. Multi-drug resistance of chemotherapeutic agents prevails as a major hindrance in breast cancer treatment [5]. Meanwhile, reports have credited the involvement of different factors for potentially influencing the chemosensitivity of tumor cells [6–8]. MicroRNA (miR) profiles in combination with other vital factors have been demonstrated to be functional in the occurrence of breast cancer [9]. Besides, a former study illustrated the association of developed resistance of breast cancer cell line MCF-7 to cisplatin with abnormal expressions of miRs and their targets [10]. In addition, it is reported that functionality of several long noncoding RNAs (lncRNAs) to be vital in tumor drug resistance [6].

LncRNAs are non-protein-coding RNAs involved in various biological processes and pathological changes [11]. The clinical significance of abnormal expression of lncRNAs in breast cancer tissues is demonstrated for the prediction of the current cancer stage and survival rate of patients with this cancer [12]. A recent study has illustrated the functionality of lncRNA UCA1 to amplify tamoxifen resistance in breast cancer cells [13]. The dysregulation of zinc finger E-box binding homeobox 1 antisense 1 (ZEB1-AS1) is credited to be of pivotal function in tumorigenesis and tumor development [14]. A prior study has observed ZEB1-AS1 to be activated in hepatocellular cancer and promotes tumor cell metastasis [15]. Furthermore, bioinformatics website (https://cm.jefferson.edu/rna22/) predicted ZEB1-AS1 to bind to miR-129-5p. MiR-129-5p has been demonstrated to stimulate cell proliferation and invasion in breast cancer [16]. Meanwhile, miR-129-5p promotes epithelial-mesenchymal transition (EMT) and regulates multi-drug resistance in breast cancer cells based on an existing study [7]. Moreover, ZEB1-AS1 exercises its oncogenic properties on osteosarcoma upon upregulation of Zinc-finger enhancer binding protein (ZEB1) [17]. A recent study ascertained ZEB1-AS1 to regulate ZEB1 expression in various types of cancers [18]. ZEB1 has been associated with breast cancer progression by promoting EMT, tumorigenesis, and angiogenesis in breast cancer [19, 20]. ZEB1 has been identified as a pivotal role in resistance to antiestrogen therapies in breast cancer treatment [8]. Hence, ZEB1 is of key importance in chemotherapeutic resistance in breast cancer therapy [21]. Overexpressed *P*-*gp* protein has been demonstrated as an essential marker for MDR in cancer cells [22]. The influence of *MDR1* and *P*-*gp* has been observed to be significant in the pharmacokinetics of many drugs, and *MDR1*-encoded-*P*-*gp* could lead to drug resistance [23, 24]. On the basis of the aforementioned literatures, we speculated the involvement of lncRNA ZEB1-AS1 in breast cancer by regulating ZEB1 and miR-129-5p. Thus, this study was conducted to explore the effects of miR-129-5p, ZEB1-AS1 and ZEB1 on drug resistance in breast cancer. These results could serve as an insight of a novel therapeutic target in breast cancer treatment.

## Methods and materials

### Ethics statement

This study was conducted under the approval of the Ethics Committee of Jiangsu Cancer Hospital, Jiangsu Institute of Cancer Research, The Affiliated Cancer Hospital of Nanjing Medical University. All patients and/or their legal guardians signed informed consent prior to participation.

### Bioinformatics prediction

The Gene Expression Omnibus (GEO) database (http://www.ncbi.nlm.nih.gov/geo) was retrieved to download chip data (GSE26910) relevant to breast cancer and annotation file of probe which were detected using the Affymetrix Human Genome U133 Plus 2.0 Array. The Affy package contained R Programming Language was employed for background correction and normalization of each chip data [25]. Based on the linear model-Empirical Bayes statistics method in the Limma package and the traditional *t*-test, nonspecific filtration of the expression data were conducted to screen the differentially expressed lncRNAs [26].

### Clinical patient samples

In total, 118 specimens with complete clinical information were acquired by the department of pathology of the Jiangsu Cancer Hospital, Jiangsu Institute of Cancer Research, The Affiliated Cancer Hospital of Nanjing Medical University from August 2014 to October 2016. All specimens including the 53 cases of invasive breast cancer, 21 cases of ductal carcinoma in situ, 22 cases of node-positive breast cancer, and 22 cases of paracancerous tissues were embedded in paraffin for storage. All samples were acquired from females including 66 cases of under 50 years old and 52 cases of over 50 years old; 36 cases with a tumor size of less than 2 cm, 82 cases with a tumor size greater than 2 cm; 47 cases without lymph node metastasis (LNM), and 71 cases with LNM. All patients had primary lesions and none of them underwent chemotherapy, radiotherapy or endocrine therapy before operation.

All of the enrolled 118 cases were interviewed by telephone or return visit during the follow-up of 7–36 months (the deadline is October 2019). The overall survival (OS) was defined as the time from randomization to death from any cause. A total of 11 were lost to follow-up and the follow-up rate was 90.68%.

### Immunohistochemistry analysis

Sections with a thickness of 4 μm were embedded separately from the normal paraffin blocks and then subjected to incubation in an oven at 60 °C for 30 min. The sections were dewaxed and hydrated successively in a conventional manner using xylene I, xylene II, 100% ethanol, 95% ethanol, 85% ethanol and 80% ethanol, 5 min for each reagent. Next, the sections were rinsed with water for 2 min, subjected to microwave antigen retrieval using 1 mM Tris-ethylene diamine tetraacetic acid (EDTA) (pH = 8.0) and cooled down to room temperature. Next, the sections were rinsed 3 times with phosphate buffer saline (PBS) (5 min for each time), incubated with 3% H_2_O_2_-methanol at room temperature for 10 min to block endogenous peroxidase, and then finally rinsed with PBS twice, 5 min each time. The primary antibody ZEB1 (ab203829, 1:100) was added to the blocks and incubated at 4 °C overnight. The next day, the sections were rinsed with 0.1% Phosphate Buffered Saline with Tween-20 (PBST) 3 times (5 min for each time), followed by the addition of polymer enhancer, and then incubated at room temperature for 20 min. Afterwards, the sections were rinsed using with 0.1% PBST 3 times (5 min for each time), incubated with the enzyme-labeled anti-rabbit/mice polymer (PV-9000-D, ZSGB-Bio, Beijing, China) at room temperature for 30 min, washed with 0.1% PBST 3 times (5 min for each time), developed using diaminobenzidine (DAB) for 5 min, and rinsed with distilled water to terminate any further development. After being counterstained with hematoxylin, the sections were rinsed with water, fully differentiated and rinsed again with water for a color change (back to blue). At last, the sections were conventionally dehydrated, cleared, and then sealed with neutral gum. A microscope (CX41, OLYMPUS Optical Co., Ltd., Tokyo, Japan) was used to observe and photograph the cover glass. In the positive cells, ZEB1 was predominantly localized in the nucleus compared to the cytoplasm. The conducted nuclear staining was concluded to be positive. ZEB1 staining in the nucleus was uneven with a focal point shape. The observation of brown or light brown nucleus was regarded as positive, while no observation of a brown or light brown nucleus was regarded as negative. A total of 5 lesion visual fields (400×) with the most intensive expression were selected on random to calculate the ratio of positive tumor cells to the total tumor cells with the mean value calculated. Cases with over 10% (including 10%) positive cells were regarded as positive, while the cases without positive staining or with positive cells less than 10% were regarded as negative.

### Cell culture

MCF-7 breast cancer cells (ATCC, Manassas, VA, USA) were incubated in Dulbecco’s modified eagle medium (DMEM) containing 10% fetal bovine serum (FBS) in a 5% CO_2_ incubator at 37 °C. MDA-MB-231 cells (ATCC, Manassas, VA, USA) were cultured in Leibovitz’s 15 medium (L15, Gibco) supplemented with 10% FBS under similar conditions. Upon observing the cell adherence, the cells were sub-cultured and treated with 0.25% trypsin. Cells in the logarithmic growth phase were chosen for subsequent experimentation.

### Fluorescent in situ hybridization (FISH)

A FISH Kit (Ribobio biotech, Guangzhou, China) was employed for in situ detection of the ZEB1-AS1 expression in MCF-7 cells. The cover glasses were placed in the hole bottom of a 24-well plate, and MCF-7 cells in the logarithmic growth phase were transferred to the cover glasses (6 × 10^4^ cells/well). When cell confluence reached 60–70%, the cells were rinsed with 1× PBS for 5 min, and fixed using 4% polyoxymethylene at room temperature for 10 min. Next, the cells were rinsed with 1× PBS, 3 times for 5 min each time. Then, 1 mL of pre-cooled permeable agent was added to all wells, and allowed to stand for 5 min at 4 °C with elimination of the permeable agent. Next, the cells were rinsed with 1× PBS, 3 times for 5 min. Afterwards, 200 μL of prehybridization solution was added into each well, and then sealed at 37 °C for 30 min. Simultaneously, the prehybridization solution was prepared by preheating at 37 °C. A total of 2.5 μL of FISH Probe Mix solution (20 μM) was added into the prehybridization solution in conditions devoid of light. After removal of the prehybridization solution from each well, cells in each well were hybridized with the hybridization solution containing probe conditions devoid of light at 37 °C overnight. Next, the cells in each well were rinsed with lotion I, 3 times (5 min for each time) at 42 °C in conditions devoid of light to reduce the background signal, and then rinsed again with lotion II once at 42 °C in similar conditions and lotion III once at 42 °C in the same environment. After a rinse with 1× PBS at room temperature in conditions devoid of light for 5 min, the cells were stained using 4′,6-diamidino-2-phenylindole (DAPI) for 10 min under similar conditions, and rinsed with 1× PBS 3 times (5 min for each time) under preexisting conditions. The cover glasses were removed from each well under conditions devoid of light, and fixed on glass slides using sealant for fluorescence detection. The specific probe of ZEB1-AS1 was synthesized by Ribobio biotech (Guangzhou, Guangdong, China).

### Dual luciferase reporter gene assay

Bioinformatics prediction website (https://cm.jefferson.edu/rna22/) was employed to analyze the binding site among miR-129-5p, ZEB1-AS1 and ZEB1, and to obtain fragment sequences containing the binding sites. ZEB1-AS1 full-length and ZEB1 3′-untranslated Region (3′UTR) region were cloned and amplified into luciferase carrier of pmirGLO (E1330, Promega, Madison, WI, USA), and named as pZEB1-AS1-wild type (Wt) and pZEB1-Wt. Based on the predicted binding sites between miR-129-5p and ZEB1-AS1, as well as miR-129-5p and ZEB1, site-specific mutagenesis was conducted. The pZEB1-AS1-mutant (Mut) and pZEB1-Mut vectors were constructed respectively, with the pRL-TK vector (E2241, Promega, Madison, WI, USA) expressing ranilla luciferase as the internal reference. MiR-129-5p mimic and miR-129-5p negative control (NC) were separately co-transfected with the luciferase reporter vector into MCF-7 cells (CRL-1415, ATCC, Manassas, VA, USA). The luminescence intensity was then detected under a fluorescence detector (Glomax20/20, ATCC, Manassas, VA, USA).

### RNA pull-down assay

A total of 50 nM biotin-labeled Wt-bio-miR-129-5p and Mut-bio-miR-129-5p were employed to transfect the MCF-7 cells. After 48 h, the cells were collected, washed with PBS, and subjected to incubation in the specific lysis buffer (Ambion, Austin, Texas, USA) for 10 min. Afterwards, the lysate was incubated with the M-280 streptomycin magnetic beads (s3762, Sigma, St. Louis, MO, USA) precoated with RNase-free bovine serum albumin (BSA) and yeast tRNA (TRNABAK-RO, Sigma, St. Louis, MO, USA). The beads were incubated at 4 °C for 3 h, and then rinsed with the pre-cooling lysis buffer twice, and then sequentially rinsed with low salt buffer 3 times and finally with high-salt buffer once. The combined RNA was purified using Trizol, and the ZEB1-AS1 expression was detected by conducting reverse transcription quantitative polymerase chain reaction (RT-qPCR).

### RNA-immunoprecipitation (RNA IP) assay

Lysis buffer [25 mM Tris-hydrochloride (HCl) (pH 7.4), 150 mM NaCl, 0.5% Nonidet P-40 (NP-40), 2 mM EDTA, 1 mM NaF and 0.5 mM dithiothreitol] containing RNasion (Takara, Tokyo, Japan) and protease inhibitor mixture (B14001a, Rochester Hills, MI, USA) were employed to split the cells. The lysate was centrifuged at 25,764×*g* for 30 min with the supernatant collected. Then the anti-Ago-2 magnetic beads (BMFA-1, BioMarker, Beijing, China) were added to the supernatant, while anti-immunoglobulin G (IgG) magnetic beads were added into the control group. After 4-h incubation at 4 °C, the washing buffer [50 mM Tris–HCl, 300 mM NaCl (pH 7.4), 1 mM MgCl_2_, and 0.1% NP-40] was employed to wash the beads 3 times. RNA was extracted from the beads using Trizol, followed by the determination of ZEB1-AS1 by RT-qPCR.

### Cell grouping and transfection

The cultured cells were classified into 12 groups: the control group (without any treatment), the NC group (transfected with empty vector), the si-ZEB1-AS1 group (transfected with si-ZEB1-AS1), miR-129-5p mimic group (transfected with miR-129-5p mimic), the miR-129-5p inhibitor group (transfected with miR-129-5p inhibitor), and the si-ZEB1-AS1 + miR-129-5p mimic group (transfected with si-ZEB1-AS1 and miR-129-5p mimic), the si-NC group (negative control of si-ZEB1), the si-ZEB1 group (transfected with si-ZEB1), the oe-NC group (transfected with empty vector), the oe-ZEB1 group (transfected with overexpressed ZEB1 plasmid), the miR-129-5p inhibitor + si-ZEB1 group (transfected with miR-129-5p inhibitor and si-ZEB1), and the miR-129-5p mimic + oe-ZEB1 group (transfected with miR-129-5p mimic and overexpressed ZEB1 plasmid). The vectors, si-ZEB1-AS1, si-ZEB1, oe-ZEB1, miR-129-5p mimic and miR-129-5p inhibitor were purchased from Ribobio (Guangzhou, Guangdong, China). Cells were inoculated into a 50 mL culture bottle with complete medium until the cell confluence reached 50–60%. Lipofectamine 2000 (Gibco, Grand Island, NY, USA) and RNA or DNA ready for transfection (5 µL lipofectamine 2000 + 100 µL serum-free culture medium placed at room temperature for 5 min; 50 nmol RNA or 2 μg DNA ready for transfection + 100 μL serum-free culture medium) were prepared in a sterile eppendorf (EP) tube. The mixture was placed at room temperature for 20 min to facilitate the complex formation of sRNA or DNA with the liposomes. The cells in the culture bottle were washed with serum-free culture medium. The complex was completely mixed with serum-free medium without penicillin/streptomycin, and then transferred to a 10 mL culturing bottle for transfection and incubation with 5% CO_2_ at 37 °C, followed by further incubation in new complete medium after 6–8 h.

### RT-qPCR

MCF-7 cells and MDA-MB-231 in the logarithmic growth phase were transfected for 48 h and then collected, followed by total RNA extraction using the MiRNeasy Mini Kit (Qiagen, Duesseldorf, Germany). A total of 5 μL RNA samples were diluted using ultrapure water without RNA enzyme 20 times. Next, the optical density (OD) value at the wavelength of 260 nm and 280 nm was detected using an ultraviolet spectrophotometer, which was followed by the determination of the concentration and purity of RNA. The OD260/OD280 ratio between 1.7 and 2.1 was reflective of high purity, which was in accordance with the requirement for subsequent experiments. According to the instructions of the reverse transcription kit (TransGene Biotech, Beijing, China), reverse transcription was conducted using a PCR thermal cycler in order to synthesize the complementary DNA (cDNA) template. The primers of ZEB1-AS1, miR-129-5p, ZEB1, B-cell lymphoma-2 (*Bcl*-*2*) and *MDR1* were designed and synthesized by Sangon Biotch (Shanghai, China) (Table 1). A total of 20 μL reverse transcription system was conducted in strict accordance with the provided instructions of EasyScript First-Strand cDNA Synthesis SuperMix (AE301-02, Transgene Biotech, Beijing, China). Subsequently, 5 μL Mix reagent, 5 μL total RNA, 1 μL random primer and 9 μL RNase Free H_2_O were added into an EP tube, centrifuged, evenly mixed to prepare a homogenous solution, and reversely transcribed in a PCR instrument (9700, Beijing Dingguochangsheng Biotechnology CO., Ltd., Beijing, China) under the following conditions: 37 °C for 15 min and 85 °C for 5 s; reaction termination at 4 °C and cDNA stored at 20 °C. The cDNA was collected for RT-qPCR following the provided instructions of the SYBR^®^*Premix Ex Taq*™ II kit (TaKaRa, Dalian, China). The reaction system was 20 μL in total, comprising of 10 μL SYBR Premix, 2 μL cDNA template, 0.6 μL forward primer, 0.6 μL reverse primer, and 6.8 μL sterilized water. Then 7500 type fluorescence quantitative PCR instrument (ABI Company, Oyster Bay, NY USA) was utilized for RT-qPCR, with *U6* as the internal reference of miR-129-5p, while glyceraldehyde-3-phosphate dehydrogenase (*GAPDH)* served as an internal reference of other genes. The reaction conditions were as follows: pre-denaturation at 95 °C for 30 s; 45 cycles of denaturation at 95 °C for 30 s, annealing for 20 s and extension at 72 °C for 30 s. Next, the expression of ZEB1-AS1, miR-129-5p, ZEB1, *Bcl*-*2* and *MDR1* was determined. The ratio of the target gene expression between the experimental group and the control group was expressed based on the 2^−ΔΔCt^ method and the formula was: ΔΔCT = ΔCt_experimental group_ − ΔCt_control group_ [27]. Ct denoted the number of amplification cycles when the real time fluorescence intensity reached the set threshold, and the amplification was denoted in the logarithmic growth phase. The experiment was repeated 3 times.

**Table 1:** Primer sequences for RT-qPCR

Genes	Sequence
U6	F: 5′-AAAGCAAATCATCGGACGACC-3′
	R: 5′-GTACAACACATTGTTTCCTCGGA-3′
GAPDH	F: 5′-TGTGGGCATCAATGGATTTGG-3′
	R: 5′-ACACCATGTATTCCGGGTCAAT-3′
ZEB1	F: 5′-ACCTCTTCACAGGTTGCTCCT-3′
	R: 5′-AGTGCAGGAGCTGAGAGTCA-3′
Bcl-2	F: 5′-GTCTTCGCTGCGGAGATCAT-3′
	R: 5′-CATTCCGATATACGCTGGGAC-3′
MDR1	F: 5′-GCCTGGCAGCTGGAAGACAAATACACAAAATT-3′
	R: 5′-CAGACAGCAGCTGACAGTCCAAGAACAGGACT-3′
miR-129-5p	F: 5′-GATCCGCAAGCCCAGACCGCAAAAAGTTTTTA-3′
	R: 5′-AGCTTAAAAACTTTTTGCGGTCTGGGCTTGCG-3′
ZEB1-AS1	F: 5′-GAGAGGCTAGAAGTTCCGCT-3′
	R: 5′-ACAAGCACCGTGTGGGTATT-3′

*F* forward, *R* reverse, *U6* small nuclear ribonucleic acid 6, *GAPDH* glyceraldehyde-3-phosphate dehydrogenase, *ZEB1* zinc finger E-box-binding homeobox 1, *Bcl-2* B-cell lymphoma 2, *MDR1* multidrug resistance protein 1, *RT-qPCR* reverse transcription quantitative polymerase chain reaction, *miR-129-5p* microRNA-129-5p, *ZEB1-AS1* zinc finger E-box binding homeobox 1 antisense 1

### Western blot analysis

MCF-7 and MDA-MB-231 cells in the logarithmic growth phase were transfected, followed by removal of the cell culture medium after 48 h. Next, the cells were rinsed with pre-cooled PBS 3 times, after which the prepared radioimmunoprecipitation assay (RNA IPA) lysis buffer (Beyotime biotechnology, Shanghai, China) was added, and scraped using a cell scratcher. The cell samples were transferred to 1.5 mL centrifuge tube and stirred using the needle 5 times for complete separation of cells. After centrifugation at 35,068×*g* for 10 min and collection of the supernatant, the protein concentration was identified following the bicinchoninic acid (BCA) method. Subsequently, the cell samples were stored at − 20 °C. The sodium dodecyl sulfate polyacrylamide gel electrophoresis (SDS-PAGE) kit was used to prepare 10% separate gel and 5% spacer gel. After electrophoretic separation on polyacrylamide gel, the protein was transferred onto a nitrocellulose (NC) membrane by wet transfer method, and sealed using 5% BSA at room temperature for 1 h. Subsequently, the NC membrane was incubated with the diluted primary antibody ZEB1 (ab203829, 1:1000), P-glycoprotein (*P*-*gp*) (ab129450, 1:2000), *Bcl*-*2* (ab59348, 1:1000), and GAPDH (ab9485, 1::2500) overnight at 4 °C. All antibodies were purchased from Abcam (Cambridge, MA, USA). The next day, the membrane was rinsed using PBST 3 times, 10 min for each time, then incubated with the secondary antibody goat-anti rabbit polyclonal antibody (ab7312, Abcam, Cambridge, MA, USA) diluted using 5% skim milk, and subjected to an oscillator at room temperature for 1 h. The membrane was rinsed using with PBST again three times (15 min each), and developed using the bio-Rad Gel Imaging System (MG8600, Beijing Thmorgan Biotechnology Co., Ltd., Beijing, China). IPP7.0 software (Media Cybernetics, Singapore) was employed for quantitative analysis. The ratio of ZEB1, *Bcl*-*2*, and *P*-*gp* to GAPDH represented their respective protein levels.

### Chemosensitivity assay

MCF-7 and MDA-MB-231 cells in the logarithmic growth phase were transfected for 48 h, detached to prepare the cell suspension, and then inoculated into a 96-well plate at a density of 1 × 10^4^ cells/well. After observation of cell adherence, the medium was replaced with medium containing variable concentrations of cisplatin (0, 2.5, 5, 10, 20, 40 μmol/L). After 48 h, 10% CCK8 was added to the cells for 2 h incubation in conditions devoid of light. The absorbance (A) at the wavelength of 450 nm was measured using a microplate reader, after which the half maximal inhibitory concentration (IC_50_) in each group was calculated. Each group comprised of set 5 duplicate wells, and the control wells without culture medium. The experiment was repeated 3 times.

### Flow cytometry

Annexin V-Fluorescein isothiocyanate (FITC)/propidium iodide (PI) double staining reagent kit (556547, Shanghai SOLJA Technology Co., Ltd., Shanghai, China) was employed to determine apoptosis of MCF-7 and MDA-MB-231 cells 48 h after transfection. The procedures were as follows: dilution of 10× binding buffer to 1× binding buffer using deionized water; centrifugation of MCF-7 cells in each group at 716×*g* at room temperature for 5 min, and cell collection. The cells were resuspended with pre-cooled 1× PBS, centrifuged at 7×*g* for 5–10 min, rinsed, and resuspended using 300 µL 1× binding buffer. Afterwards, the cells were thoroughly mixed 5 µL Annexin V-FITC and incubated at room temperature for 15 min in conditions devoid of light. Next, 5 µL PI was added to the cells 5 min before conducting the flow cytometry detection (Cube6, Partec, Germany), and ice-bathed under conditions void of light for 5 min. FITC was detected at excitation wavelengths of 480 nm and 530 nm, and PI was detected at an excitation wavelength over 575 nm.

### Statistical analysis

The SPSS 21.0 software (IBM Corp., Armonk, NY, USA) was employed for statistical analysis. Measurement data were expressed by mean ± standard deviation. Data between two groups were compared by unpaired *t*-test, while comparison among multiple groups was analyzed by one-way analysis of variance (ANOVA), followed by Tukey’s post hoc test. Kaplan–Meier analysis was used to analyze the correlation between the ZEB1 expression and the OS rate of patients, and analysis of the differences was performed by the log-rank test. The clinicopathological data of all participants were enumeration data, which were expressed by cases and percentage and analyzed by Chi-square test. A value of *p* < 0.05 was indicative of a statistically significant difference.

## Results

### ZEB1-AS1 is overexpressed in breast cancer and mainly locates in cytoplasm

Microarray analysis was employed to screen out differentially expressed lncRNA. Results revealed that ZEB1-AS1 was highly expressed in breast cancer (Fig. 1a). Besides, FISH was conducted to determine the location of ZEB1-AS1 in MCF-7 cells, and the results showed that ZEB1-AS1 was predominantly expressed in the cytoplasm (Fig. 1b). Thus, based on the evidence it can be concluded that ZEB1-AS1 was expressed highly in breast cancer and principally localized in the cytoplasm.

**Fig. 1:** ZEB1-AS1 is highly expressed with a predominant expression in the cytoplasm (400×). **a** RCicos of breast cancer-related chip GSE26910; **b** subcellular localization of ZEB1-AS1 (400×); DAPI referred to localization of nucleus, Inc showed the localization of ZEB1-AS1, and merge displayed the combined results of DAPI and Inc; *ZEB1-AS1* zinc finger E-box-binding homeobox 1-antisense 1

### ZEB1-AS1 may regulate ZEB1 by competitively binding to miR-129-5p

Dual luciferase reporter gene assay, RNA IP and RNA pull-down were employed to determine the interactions among ZEB1-AS1, ZEB1 and miR-129-5p. The online prediction software suggested the existence of various binding sites between miR-129-5p and ZEB1 3′UTR region, as well as miR-129-5p and ZEB1-AS1. In comparison with the NC group, the luciferase activity in the 3′UTR of ZEB1-Wt was inhibited by miR-129-5p (*p* < 0.05), whereas the luciferase activity of mutant was not affected. These results indicated that miR-129-5p specifically bound to ZEB1 3′UTR and downregulated ZEB1 gene expression after transcription (Fig. 2a). Meanwhile, the luciferase activity in the binding site between the ZEB1-AS1-Wt and miR-129-5p was inhibited by miR-129-5p, with no effect on the mutant inhibition. The results revealed that miR-129-5p could specifically bind to ZEB1-AS1 (Fig. 2b). RNA pull-down assay revealed that Wt-miR-129-5p-targeted ZEB1-AS1 was significantly increased (*p* < 0.05) compared with Mut-miR-129-5p. It suggested that miR-129-5p directly binds to ZEB1-AS1 (Fig. 2c). According to Ago2 RNA IP, Ago2 targeted-ZEB1-AS1 was obviously increased (*p* < 0.05), compared with IgG. These results indicated that ZEB1-AS1 could bind to the Ago2 protein (Fig. 2d). These results led to the speculation that ZEB1-AS1 could regulate ZEB1 by competitively binding to miR-129-5p.

**Fig. 2:** ZEB1 and ZEB1-AS1 are the target genes of miR-129-5p. **a** Verification of the target relationship between miR-129-5p and ZEB1 by dual luciferase reporter gene assay; **b** identification of the target relationship between miR-129-5p and ZEB1-AS1 by dual luciferase reporter gene assay; **c** determination of relative ZEB1-AS1 enrichment by RNA pull-down; **d** determination of relative ZEB1-AS1 enrichment by RNA IP; * indicates *p* < 0.05 vs. the control group or IgG group. *ZEB1-AS1* zinc finger E-box-binding homeobox 1-antisense 1, *ZEB1* zinc finger E-box-binding homeobox 1, *WT* wild type, *MUT* mutant, *miR* microRNA, *IgG* immunoglobulin G, *Ago2* argonaute2

### Overexpressed miR-129-5p or silenced ZEB1-AS1 decreases ZEB1, *Bcl*-*2*, *MDR1*, ZEB1-AS1 expression, yet increases expression of miR-129-5p

Primarily, RT-qPCR was conducted to determine the expression of ZEB1-AS1, miR-129-5p, ZEB1, *Bcl*-*2*, and *MDR1* in breast cancer cell lines MCF-7 and MDA-MB-231. In addition, Western blot analysis was employed to determine the protein levels of ZEB1, *Bcl*-*2* and *P*-*gp*. In comparison with the control group, no obvious change was evident in the expression of ZEB1-AS1, miR-129-5p, *Bcl*-*2*, *MDR1* and ZEB1 in the NC group; in the miR-129-5p inhibitor group, the expression of ZEB1-AS1, *Bcl*-*2*, *MDR1* and ZEB1 was increased but that of miR-129-5p was decreased; the miR-129-5p mimic and si-ZEB1-AS1 groups exhibited reduced expressions of ZEB1-AS1, *Bcl*-*2*, *MDR1* and ZEB1, yet increased expressions of miR-129-5p; the si-ZEB1-AS1 + miR-129-5p mimic group demonstrated the lowest expression of ZEB1-AS1, ZEB1, *Bcl*-*2* and *MDR1*, while the highest expression of miR-129-5p (*p* < 0.05, Fig. 3a, b).

**Fig. 3:** miR-129-5p overexpression or ZEB1-AS1 silencing decreases the expression profiles of ZEB1-AS1, *Bcl*-*2*, *MDR1* and ZEB1 but increases that of miR-129-5p. **a** Relative expression of related genes in ZEB1-AS1/miR-129-5p/ZEB1 axis in MCF-7 cell line determined by RT-qPCR; **b** relative expression of related genes in ZEB1-AS1/miR-129-5p/ZEB1 axis in MD-MB-231 cell line determined by RT-qPCR; **c** protein expression level of related genes in ZEB1-AS1/miR-129-5p/ZEB1 axis in MCF-7 cell line measured by western blot; **d** protein expression level of related genes in ZEB1-AS1/miR-129-5p/ZEB1 axis in MD-MB-231 cell line measured by western blot; * indicates *p* < 0.05 vs. the control group; *ZEB1-AS1* zinc finger E-box-binding homeobox 1-antisense 1, *ZEB1* zinc finger E-box-binding homeobox 1, *miR-129-5p* microRNA-129-5p, *Bcl*-*2* B cell lymphoma/lewkmia-2, *MDR1* multidrug resistance, *RT-qPCR* reverse transcription quantitative polymerase chain reaction

Western blot analysis ascertained no evident change in the protein levels of ZEB1, *Bcl*-*2*, and *P*-*gp* in the NC group compared with the control group; the protein levels of ZEB1, *Bcl*-*2*, and *P*-*gp* were increased in the miR-129-5p inhibitor group while they decreased in the miR-129-5p mimic and si-ZEB1-AS1 groups. The si-ZEB1-AS1 + miR-129-5p mimic group exhibited the least protein levels of ZEB1, *Bcl*-*2* and *P*-*gp* among the 6 groups (*p* < 0.05, Fig. 3c, d). These results revealed that upregulation of miR-129-5p or downregulation of ZEB1-AS1 could inhibit ZEB1, *Bcl*-*2*, *MDR1*, ZEB1-AS1, and *P*-*gp* expression, but stimulate miR-129-5p expression.

### Upregulated miR-129-5p or downregulated ZEB1-AS1 contributes to inhibited drug resistance to cisplatin in breast cancer

CCK8 was applied to detect drug resistance to cisplatin in breast cancer after transfection in breast cancer cell lines MCF-7 and MDA-MB-231. In comparison with the control group, no obvious change was evident for resistance to cisplatin in the NC group (*p* > 0.05); the resistance to cisplatin was decreased in the si-ZEB1-AS1 and mi-129-5p mimic groups, and the resistance to cisplatin in the si-ZEB1-AS1 + miR-129-5p mimic group was the lowest among all groups (*p* < 0.05). Meanwhile, the resistance to cisplatin in the miR-129-5p inhibitor group was increased significantly compared with the control group (*p* < 0.05, Table 2). Conjointly, the resistance to cisplatin decreased due to the overexpression of miR-129-5p and silencing of ZEB1-AS1.

**Table 2:** Resistance to cisplatin in each group and in two breast cell lines

Groups	MCF-7	MDA-MB-231
	IC50 (μmol/L)	IC50 (μmol/L)
Control	12.52 ± 1.17	14.63 ± 1.27
NC	13.12 ± 1.34	15.24 ± 1.31
si-ZEB1-AS1	7.89 ± 0.87*	6.57 ± 0.83*
miR-129-5p mimic	8.64 ± 0.94*	5.38 ± 0.75*
miR-129-5p inhibitor	19.65 ± 1.65*	22.84 ± 1.49*
si-ZEB1-AS1 + miR-129-5p mimic	4.06 ± 0.42*	2.26 ± 0.41*

*NC* negative control, *miR-129-5p* microRNA-129-5p, *ZEB1-AS1* zinc finger E-box binding homeobox 1 antisense 1

*p < 0.05 vs. the control group

### Upregulated miR-129-5p or downregulated ZEB1-AS1 induces cell apoptosis of breast cancer cells

Flow cytometry was employed to determine cell apoptosis in breast cancer cell lines MCF7 and MDA-MB-231. In comparison with the control group, no obvious change was evident for cell apoptosis in the NC group (*p* > 0.05), and the apoptosis rates in the si-ZEB1-AS1, miR-129-5p mimic, and si-ZEB1-AS1 + miR-129-5p mimic groups were evidently increased (*p* < 0.05), which was highest in the si-ZEB1-AS1 + miR-129-5p mimic group (*p* < 0.05); while the miR-129-5p inhibitor group showed a decreased apoptosis rate (*p* < 0.05, Fig. 4). On the basis of aforementioned evidence, it can be concluded that the overexpressed miR-129-5p or silenced ZEB1-AS1 contributed to a promotion on cell apoptosis of breast cancer cells.

**Fig. 4:** miR-129-5p upregulation or ZEB1-AS1 downregulation increases cell apoptosis in breast cancer cells. **a** Cell apoptosis of MCF-7 cells in each group; **b** statistical results of MCF-7 cell apoptosis rate of each group; **c** cell apoptosis of MDA-MB-231 cells in each group; **d** statistical results of MDA-MB-231 cell apoptosis rate of each group; * indicates *p* < 0.05 vs. control group; *NC* negative control, *ZEB1-AS1* zinc finger E-box-binding homeobox 1-antisense 1, *miR-129-5p* microRNA-129-5, *FITC* fluorescein isothiocyanate, *MCF-7* human breast adenocarcinoma cell line

### ZEB1 is associated with tumor progression and poor prognosis in patients with breast cancer

Immunohistochemistry was performed to determine ZEB1 positive expression in breast cancer tissues. Figure 5a displayed the different expression of ZEB1 in breast tissues: negative (−), weak positive (+), moderate positive (++), and strong positive (+++). Then, immunohistochemistry showed that the ZEB1 positive rates in invasive breast cancer, ductal carcinoma in situ, node-positive breast cancer and paracancerous tissues were 32.1%, 0.0%, 40.9% and 4.5%, respectively (Fig. 5b). No correlation between the ZEB1 expression and age and tumor size was evident; however, it was related with LNM (*p* < 0.05) (Table 3). Moreover, Kaplan–Meier method was employed to calculate the OS rate of patients, which revealed that patients with positive expression of ZEB1 exhibited a lower OS rate, suggesting that positive expression of ZEB1 may be associated with poor prognosis of patients with breast cancer (Fig. 5c). Thus, we conclude that ZEB1 was overexpressed and correlated with LNM and poor prognosis in breast cancer.

**Fig. 5:** Immunohistochemical detection of ZEB1 positive expression profile in four different breast cancer tissues. **a** Immunohistochemical images of different ZEB1 expression in breast tissues; negative (−), weak positive (+), moderate positive (++), and strong positive (+++); **b** immunohistochemical images of ZEB1 positive expression profile in four kinds of different breast tissues (infiltrating breast cancer, ductal carcinoma in situ, node-positive breast cancer, and paracancerous tissues); **c** the OS rate of patients with negative expression or positive expression of ZEB1 by Kaplan–Meier analysis

**Table 3:** The clinicopathological features and the expression of ZEB1 in patients with breast cancer

Clinicopathological feature	ZEB1		Cases	χ^2^	*p*
	Positive	Negative			
Age					
< 50	52 (78.8%)	14 (21.2%)	66	0.237	0.627
≥ 50	39 (75.0%)	13 (25.0%)	52		
Tumor size					
< 2 cm	29 (80.6%)	7 (19.4%)	36	0.347	0.556
≥ 2 cm	62 (75.6%)	20 (24.4%)	82		
LNM					
No	41 (87.2%)	6 (12.8%)	47	4.529	0.003
Yes	50 (70.4%)	21 (29.6%)	71		
Infiltrating breast cancer	36 (67.9%)	17 (32.1%)	53	6.460	0.011
Ductal carcinoma in situ	21 (100.0%)	0 (0.0%)	21	0.977	0.323
Node-positive breast cancer	13 (67.9%)	9 (40.9%)	22	8.282	0.004
Paracancerous tissues	21 (95.5%)	1 (4.5%)	22		

*LNM* lymph node metastasis, *ZEB1* zinc-finger E-box binding homeobox

### ZEB1 silencing inhibits MCF-7 cell resistance to cisplatin and promotes apoptosis

In order to discuss the effect of ZEB1 on the sensitivity of MCF-7 to cisplatin and apoptosis, RNA silencing and gene overexpression via plasmid were conducted. Western blot was applied to determine ZEB1, Bcl-2 and P-gb protein level (Fig. 6a), CCK-8 was used to detect drug resistance (Fig. 6b) and flow cytometry was employed to measure cellular apoptosis rate (Fig. 6c). The results showed that ZEB1, Bcl-2 and P-gb protein level increased, the cisplatin resistance raised and apoptosis decreased in the oe-ZEB1 group compared with the on-NC group. Furthermore, in contrast to the si-NC group, the ZEB1, Bcl-2 and P-gb protein levels decreased as well as cisplatin resistance; however the apoptosis was significantly elevated in the si-ZEB1 group. A combination of miR-129-5p mimic with oe-ZEB1 reduced ZEB1, Bcl-2 and P-gb expressions, decreased MCF-7 cisplatin resistance and elevated cell apoptosis. Instead, the effects were reversed in the miR-129-5p inhibitor and si-ZEB1 group compared with the si-ZEB1 group. Therefore, it can be concluded that the regulation of MCF-7 sensitivity and apoptosis was mediated by ZEB1.

**Fig. 6:** Regulation of ZEB1 expression affects cisplatin resistance and apoptosis of MCF-7. **a** Detection of ZEB1, Bcl-2 and P-gb protein level in the breast cancer cell line MCF-7 via western blot; **b** detection of the cisplatin sensitivity of MCF7 cell line; **c** measurement of MCF-7 apoptosis by flow cytometry. * indicates *p* < 0.05 vs. the control group; *ZEB1-AS1* zinc finger E-box-binding homeobox 1-antisense 1, *ZEB1* zinc finger E-box-binding homeobox 1, *miR-129-5p* microRNA-129-5p, *oe* overexpression

## Discussion

Breast cancer is a heterogeneous disease presenting with a poor prognosis due to variations in the biological characters and clinical response [28, 29]. Currently, tumor drug resistance prevails to be problematic for attaining successful chemotherapeutic results in breast cancer [30]. Recent evidence has suggested the involvement of lncRNAs in tumor drug resistance, which could provide an insight for overcoming drug resistance in cancer treatment [6]. Therefore, the aim of our study was to evaluate the effect of lncRNA ZEB1-AS1 on drug resistance in breast cancer. Collectively, our data from the present study revealed that that restraint of ZEB1-AS1 exercises its inhibitory role in drug resistance in breast cancer via up-regulating miR-129-5p and down-regulating ZEB1.

Initially, based on our findings, lncRNA ZEB1-AS1 and ZEB1 exhibited elevated expressions in breast cancer cells. A recent study has demonstrated that expression of lncRNA ZEB1-AS1 to be up-regulated in osteosarcoma, which could potentially accelerate osteosarcoma occurrence rate [31]. Another study has confirmed that lncRNA ZEB1-AS1 is highly expressed in hepatocellular cancer tissues, predominantly in metastatic cancerous tissues, which corresponds with the high mortality and morbidity among patients with hepatocellular cancer [15]. Evidence has suggested a correlation between overexpressed ZEB1 and unsatisfactory prognosis of various malignancies, including breast cancer [32]. The observation of an up-regulated ZEB1 expression has been frequent in breast cancer tissues in contrast with benign tissues related to breast disease and its up-regulation is associated with lymph node metastasis, the size of tumor and elevated tumor stage in breast cancer [33]. Conjointly, the aforementioned findings were consistent with our observation of high levels of lncRNA ZEB1-AS1 and ZEB1 in breast cancer cells.

Additionally, by means of the target prediction program and the dual luciferase activity determination, our study demonstrated that ZEB1-AS1 regulated the expression of ZEB1 by competitively binding to miR-129-5p. LncRNA ZEB1-AS1 has been proven to promote cell metastasis via upregulation of ZEB1 in hepatocellular cancer based on a recent study [34]. Besides, another study has ascertained the involvement of miRs in tumor progression and invasion through interaction with target genes within cells [35]. Notably, a correlation has been reported previously between lncRNA MALAT1 silencing and the inhibition of cell migration, invasion and proliferation in triple-negative breast cancer through regulation of miR-129-5p [16]. Furthermore, consistent with our results, an existing study has revealed that miR-129-5p silencing increased ZEB1 expression in breast cancer MCF-7 cells [36]. Collectively, the aforementioned provided further evidence to substantiate our result supporting the functionality of ZEB1-AS1 as a regulator in ZEB1 expression by competitively binding to miR-129-5p.

Moreover, our findings also proved that overexpressed miR-129-5p or silenced ZEB1-AS1 contributed to the decreased expressions of ZEB1, *Bcl*-*2, MDR1*, *P*-*gp* and ZEB1-AS1, thus reducing drug resistance to cisplatin and enhancing the overall cell apoptosis in breast cancer. An existing study has reported ZEB1-AS1 to exercise a stimulative effect on osteosarcoma development by activating ZEB1 and its knockdown could potentially suppress cell migration and proliferation in osteosarcoma [17]. Moreover, the functionality of *Bcl*-*2* has been ascertained as a key regulator along the apoptotic process [37]. A previous study demonstrated that miR-34a overexpression attenuated cell proliferation and migration which critically enhanced apoptosis in breast cancer by decreasing *Bcl*-*2* expression [38]. Besides, the functionality ZEB1 has been confirmed as a stimulant for increasing *Bcl*-*2* expression [39]. Meanwhile, suppressed expressions of the *MDR1*, and *P*-*gp* gene as well as drug resistance have been evidently detected among breast cancer patients undergoing treatment with glucosylceramide synthase [40]. Another existing study revealed that miR-129 overexpression inhibits cisplatin-resistance in human gastric cancer cells by inhibiting *P*-*gp*, which is in consistency with our results [41]. Moreover, our findings illustrated upregulated miR-129-5p and downregulated ZEB1-AS1 to potentially promote cell apoptosis in breast cancer. Consistent with our results, a recent study revealed that ZEB1-AS1 knockdown could efficaciously restrain cell proliferation and induce cell apoptosis in colorectal cancer [42].

Finally, through the treatment of ZEB1 silence and overexpression in MCF-7 cell line, the role of microRNA-129-5p and ZEB1 in the cisplatin resistance of MCF-7 cells was evaluated. Reports have demonstrated the involvement of ZEB1 with cisplatin resistance in ovarian cancer [43], stomach cancer [44] and non-small cell lung cancer (NSCLC) [45]. Moreover, the downstream genes regulated by ZEB1 include ABCG2 and ERCC1 in NSCLC [46] as well as SLC3A2 in ovarian cancer [43]. Therefore we speculated that these targeted genes might participate in drug resistance of breast cancer, which requires further investigation.

## Conclusion

The findings from this study revealed that ZEB1-AS1 silencing down-regulated ZEB1 by elevating miR-129-5p, thus decreasing drug resistance to cisplatin and promoting cell apoptosis in breast cancer, which might serve as the theoretical foundation for the development of new therapeutic targets and provide potential tumor chemosensitizer in breast cancer treatment. However, due to the limitations on time, space and study subjects, this study was not so comprehensive and might be inadequate to substantiate theoretical basis. Thus, additional statistics are necessary for more credible results, and further studies are expected to explore whether ZEB1 is the sole transcription factor related to drug resistance in breast cancer, as well as the regulatory mechanism responsible for miRNA-129-5p on ZEB1.

## Data Availability

The datasets generated/analysed during the current study are available.

## Abbreviations

lncRNA: Long non-coding RNA
miR-129-5p: microRNA-129-5p
GEO: Gene Expression Omnibus
LNM: Lymph node metastasis
PBS: Phosphate buffer saline
PBST: Phosphate Buffered Saline with Tween-20
DAB: Diaminobenzidine
FBS: Fetal bovine serum
FISH: Fluorescent in situ hybridization
NC: Negative control
BSA: Bovine serum albumin
